RETRACTED

# Delicaflavone Represses Lung Cancer Growth by Activating Antitumor Immune Response through N6-Methyladenosine Transferases and Oxidative Stress

**DOI:** 10.1155/2022/8619275

**Published:** 2022-08-08

**Authors:** Xuewen Wang, Dafen Xu, Bing Chen, Dandan Huang, Zhijun Li, Yuxia Sui, Fei Lin, Hong Yao, Huang Yuan Li, Xinhua Lin

**Affiliations:** ^1^Department of Preventive Medicine, School of Public Health, Fujian Medical University, Fuzhou 350122, China; ^2^Department of Pharmaceutical Analysis, School of Pharmacy, Fujian Medical University, Fuzhou 350122, China; ^3^Key Laboratory of Nanomedical Technology (Education Department of Fujian Province), School of Pharmacy, Nano Medical Technology Research Institute, Fujian Medical University, Fuzhou 350122, China; ^4^School of Pharmacy, Fujian Medical University, Fuzhou, 350122 Fujian, China; ^5^Department of Pharmacy, Shengli Clinical Medical College of Fujian Medical University, Fuzhou 350001, China; ^6^Department of Pharmacy, Fujian Provincial Hospital, Fuzhou 350001, China; ^7^Fujian Key Laboratory of Drug Target Discovery and Structural and Functional Research, Fujian Medical University, Fuzhou 350122, China; ^8^Fujian Provincial Key Laboratory of Environment Factors and Cancer, School of Public Health, Fujian Medical University, Fuzhou 350122, China

## Abstract

Our previous studies have shown that delicaflavone (DLL), a biocomponent extracted from *Selaginella doederleinii* Hieron, has antitumor activity. However, the role of DLL in the antitumor immune response is unknown. In this study, we tested the potential roles of DLL in antitumor immune response. An animal tumor model with Lewis lung cancer cell line (3LL) in C57BL/6 mice was established to determine whether DLL induced the tumor-bearing host's antitumor immune response. m6A-MeRIP-qPCR, western blot, and flow cytometry were performed to explore the underlying mechanisms. DLL inhibited the proliferation of 3LL lung cancer cells *in vitro* and *in vivo* and induced tumor cell oxidative stress. DLL significantly inhibited tumor growth in immunocompetent mice compared with nude mice. DLL treatment significantly increased Th1 cytokine production and CD8+ T cell infiltration into tumor tissues in tumor-bearing mice. DLL-mediated antitumor immune effects were reversed by overexpression of the N6-methyladenosine (m6A) transferase Mettl3/Mettl14. Mechanistically, DLL upregulated the expression of Stat1 and Irf1 and the secretion of cytokines by inhibiting Mettl3 and Mettl14 in lung cancer cells. In conclusion, DLL inhibited lung cancer cell growth by suppressing Mettl3/Mettl14 to activate antitumor immunity. These findings provided an opportunity to enhance lung cancer immunotherapy.

RETRACTED

## 1. Introduction

Traditional Chinese medicines have distinct advantages in tumor treatments [1]. They fight cancer by inducing tumor cell apoptosis, inhibiting tumor angiogenesis, reversing multidrug resistance, and regulating the host's immune response [2].

Many biflavonoids have been found to have antitumor activity in recent studies. Natural biflavonoids are widely present in vascular plants such as *Selaginella*. *Selaginella doederleinii* Hieron has a unique antitumor effect and is commonly used clinically to treat nasopharyngeal, esophageal, gastric, liver, lung, choriocarcinoma, and cervical cancer [3]. Lee et al. found that amentoflavone significantly inhibited fatty acid synthase activity, thereby inhibiting tumor cell growth [4]. We previously isolated a new type of biflavonoid compound, delicaflavone (DLL), from *Selaginella doederleinii* Hieron, and discovered that DLL inhibited A549 cell growth via the Akt/mTOR/p70S6K signaling pathway [5]. DLL reduced cisplatin resistance in lung cancer by modulating endoplasmic reticulum stress signaling [6]; however, it is unknown whether DLL can activate an antitumor immune response.

Traditional Chinese medicine has been shown in studies to have antitumor activity via oxidative stress and epigenetic mechanisms, such as RNA methylation [7–9]. Reactive oxygen species (ROS) are known to regulate every step of tumorigenesis by acting as second messengers in cancer cells, which play essential roles in the regulation of cancer progression [10]. Traditional Chinese medicine-induced oxidative stress can regulate N6-methyladenosine (m6A) modification [11]. The interaction of m6A modification and oxidative stress influences tumor growth [12, 13]. m6A modification is an important posttranscriptional modification process that regulates mRNA localization, transcription, and stability [14]. The factors involved in m6A methylation are mainly related to three protein families: methyltransferases (writer) including METL3, METL14, and WTAP; m6A demethylases (eraser) including FTO and ALKBH5; and m6A “readers” including YTHDCs, YTHDFs, and IGF2BPs [15]. Recent research has revealed that m6A plays a role in regulating the tumor immune microenvironment [16]. Increased RNA methylation, for example, reduces the sensitivity of melanoma cells to anticancer immunotherapy [17]. ALKBH5 knockout altered the composition of tumor-infiltrating Treg cells, resulting in changes in the tumor microenvironment [18]. METTL3/14 regulates the immune response of refractory colorectal cancer anti-PD-1 treatment [19]. However, it is still unknown whether DLL can influence tumor immune response via m6A modification and oxidative stress.

RETRACTED

In this study, we tested the potential roles of DLL in antitumor immune response by establishing a lung cancer model (3LL).

## 2. Experimental Procedures

### 2.1. Cell Count Kit 8 Assay

The murine Lewis lung cancer cell line (3LL) was purchased from ATCC (USA) and was cultured in DMEM medium. The medium was supplemented with 10% FBS (fetal bovine serum).

The cell counting kit 8 (CCK-8) cell proliferation kit (cat no. CA1210, Solarbio, Beijing, China) was used for measure the inhibitory effects of DLL on 3LL cells according to the manufacturer's instructions. 3LL cells were cultured on a 96-well plate at a density of 2000 cells/well. After 24 hours of culture, the cells were exposed to different doses of DLL (0, 5, 25, 50, and 100 mg/ml) for 24, 48, or 72 hours. Then, 10 *μ*l of the CCK-8 reagent was added for 2-hour incubation at 37°C. The 450 nm absorbance was recorded.

### 2.2. Mice

C57BL/6 mice (male, 6 weeks, 18-20 g) and nude mice (male, 6 weeks, 18-20 g) were purchased from the Shanghai Experimental Center of the Chinese Academy of Sciences. Animal experiments were ethically approved by the Experimental Animal Ethics Committee of Fujian Medical University.

### 2.3. Construction of Tumor-Bearing Mice and DLL Treatment

Nude mice or immunocompetent C57BL/6 mice were randomly divided into the DLL group (*n* = 6) and the control group (treated with equal volume saline, *n* = 6). Nude mice or immunocompetent C57BL/6 mice were injected subcutaneously with 5 × 10^4^ 3LL tumor cells (day 0). On day 4, mice in the DLL group were injected with DLL (0.5 mg/kg/day, s.c.) into the subcutaneous tumors, once a day, for a total of 7 times [6]. The tumor size was measured every 2 days to monitor tumor growth in mice.

### 2.4. In Vivo Anti-IFN-*γ* Processing

Four days after subcutaneous injection of 3LL lung tumor cells, DLL was administrated intraperitoneally (0.5 mg/kg) into mice once a day, and anti-IFN-*γ* antibody (250 *μ*g) was intraperitoneally injected once a day for 7 times [20].

### 2.5. Flow Cytometry

Immune cells were stained with antibodies (anti-CD3, anti-CD4, and anti-CD8, Abcam, USA) for 30 min at 4°C. The Fixation & Permeabilization Kit (Southern Biotech, Birmingham, USA) was used for staining intracellular IFN-*γ*, IL-4, and Foxp3. The fluorescence was determined on BD FACSAria Fusion and analyzed with FlowJo software (v10.8) (Becton, Dickinson and Company, Ashland, OR, USA).

### 2.6. Sorting T Cells

The Dynabeads Untouched Mouse T Cells kit (Life Technologies) was used for isolating T cells from spleen and lymph nodes according to the manufacturer's instructions. The purified T cells were cultured in a 24-well plate. Effector T cells were activated by CD3*ε*/28.

RETRACTED

### 2.7. Lentiviral Transfection

To overexpress METTL3 and METTL14 in 3LL cells, lentiviral particles were constructed by Guangzhou Ribo Biological Company (Guangzhou, China). When the cell confluence reached about 80% in a 12-well culture plate, 3LL cells were infected with lentiviral in a 50 multiplicity of infection (MOI) value for 48 h and used for further experiments. The cells infected with negative control virus were used as control.

### 2.8. T Cell Proliferation Test In Vitro

To test the ability of T cells in killing tumor cells, the purified mouse T cells and the treated 3LL cells were cocultured at a ratio of 1 : 10 for 4 days. The BrdU Cell Proliferation ELISA kit (cat no. ab126556, Abcam) was used to access T cell proliferation in vitro according to the manufacturer's instructions. The data is expressed as the percentage of response T cell proliferation.

### 2.9. Real-Time Quantitative Polymerase Chain Reaction (qPCR)

Total RNA was extracted from cells after DLL treatment or transfection using TRIzol. cDNA was then synthesized using Superscript II (ThermoFisher), and qPCR was performed using ChamQ SYBR qPCR Master Mix (cat no. Q311-02, Vazyme, Nanjing, China). The primers are shown in Supplementary Table 1. qPCR was performed as follows: reverse transcription stage: 42°C for 10 min, initial denaturation: 95.0°C for 3 min, denaturation and extension: 38 circles of 95.0°C for 10 s and 60°C for 30 s, and melting curve analysis: 72°C-95.0°C with heating rate 0.5°C/unit time.

### 2.10. Commercial Kits

The Mouse IFN gamma ELISA Kit (ab282874, Abcam), RANTES ELISA Kit (CCL5) (ab100739, Abcam), CXCL9 ELISA Kit (ab203364), IP-10 ELISA Kit (CXCL10), SOD Kit (S0101S, Beyotime, Shanghai), NAD+/NADH Assay Kit (S0175, Beyotime, Shanghai), ATP Assay Kit (S0026, Beyotime, Shanghai), and total Glutathione Peroxidase Assay Kit (S0058, Beyotime, Shanghai) were used for supernatant analysis of the levels of IFN-*γ*, CCL5, CXCL9, CXCL10, SOD, and Gpx according to the manufacturer's instructions.

#### 2.10.1. Measurement of ROS

Briefly, after DLL treatment, 3LL cells were collected and incubated with ROS indicator DCFH-DA (10 *μ*M) in PBS for 30 min at 37°C. The fluorescence was captured and analyzed using an Accuri C6 plus flow cytometer (BD Biosciences, CA).

### 2.11. Western Blotting

After the indicated treatment, total proteins were extracted using cold RIPA buffer, and the concentrations were determined using a BCA Protein Quantification Kit (cat no. E112-01, Vazyme, Nanjing, China). The protein was separated on SDS-PAGE gel (10%) and transferred to a nitrocellulose membrane. The membranes were blocked with 5% nonfat milk and then incubated with primary antibodies (anti-METTL3, cat no. ab195352; anti-METTL14, cat no. ab220030; anti-stat1, cat no. ab109320; anti-Irf1, cat no. ab243895; anti-STAT1 (phospho S727), cat no. ab278718; and anti-GAPDH, cat no. ab8245. All the antibodies were purchased from Abcam, USA) incubated overnight at 4°C. The next day, after washing with PBS, the membranes were incubated with secondary antibody for 2 h. The positive signal was captured in the gel imaging system. The bands of western blot were quantified by ImageJ, and the relative protein expression was expressed as the optical density of bands.

RETRACTED

### 2.12. m6A Methylated RNA Immunoprecipitation Sequencing (MeRIP) qPCR

A FastPure Cell/Tissue Total RNA Isolation Kit (Vazyme, Nanjing, China) was used to extract total RNA. The RNA was incubated with A/G immunomagnetic beads and m6A antibody premix overnight at 4°C. The bounding RNA were eluted from the magnetic beads by adding 30 microliters of RLT buffer. The expression of Stat1 and Irf1 was analyzed by qPCR.

### 2.13. Immunohistochemistry

The paraffin-embedded slides in mouse tumor tissues were deparaffinized and antigen retrieved. After blocking with 5% goat serum (cat no. 5425S, Beyotime, Shanghai, China), the sections were incubated with the primary antibody anti-CD8 (Abcam, ab209775) overnight at 4°C. The sections were incubated with secondary goat anti-mouse IgG antibody (Abcam, ab205719) for 1 h. A DAB Horseradish Peroxidase Color Development Kit was used for staining the positive signals and then counterstained with hematoxylin.

### 2.14. Statistical Analysis

All experiments were independently performed three times, and the data were shown as the mean ± standard deviation (mean ± SD, *n* = 6). GraphPad Prism software was used for statistical analysis. *P* < 0.05 was statistically significant.

## 3. Results

### 3.1. DLL Significantly Inhibits Tumor Growth in Immunocompetent Mice

3LL cells were exposed to DLL (0, 5, 25, 50, and 100 *μ*g/ml). We observed that DLL inhibited 3LL cell viability in a time- and dose-dependent manner (Figure 1(a)). We next injected 3LL cells into immunodeficient nude mice. Four days after injection, DLL (0.5 mg/kg) was administrated into the tumor site every day for 7 days, and the tumor volumes were detected every two days. Interestingly, the tumor growth of nude mice treated with DLL temporarily slowed down from the 10th to 14th days, but the growth rate increased in the next 10 days (Figure 1(b)), suggesting that DLL not only directly exhibited the antitumor effect on tumor cells but also inhibited tumor cell growth through tumor microenvironment. Next, we injected 3LL cells into the immunocompetent mice (C57BL/6), administrated DLL (0.5 mg/kg) every day for 7 days, and measured tumor volume every two days. Surprisingly, DLL significantly reduced tumor volume in immunocompetent mice compared with nude mice. The tumor almost disappeared on the 16th day in DLL-treated immunocompetent mice (Figure 1(c)). These findings indicate that DLL exhibited the antitumor effect via the host immune system.

RETRACTED

### 3.2. DLL Slightly Reduces the Percentage of CD8+ T Cells in Naive Mice

We tested the roles of DLL on immune response. DLL treatment has no effects on the percentage of CD3+/CD4+ T cells and regulatory T cells. Interestingly, DLL treatment reduced the percentage of CD3+/CD8+ T cells (Figures 2(a) and 2(b)). In addition, DLL treatment significantly reduced the percentage of CD8+/IFN-*γ*+ cells, while having no effect on the percentage of CD4+/IL4+ T cells and CD4+/IFN-*γ*+ T cells (Figures 2(a) and 2(b)). These results revealed that DLL treatment mildly suppressed the initial immune response.

### 3.3. DLL Treatment Increases the Percentage of CD8+ T Cells in Tumor-Bearing Mice

We next investigated the alterations of immune patterns in DLL-treated immunocompetent tumor-bearing mice. DLL treatment significantly increased the percentage of CD3+ T cells and CD8+ T cells in the lymph nodes and spleen and mildly decreased the percentage of Treg T cells (Figures 3(a) and 3(b)). In addition, DLL treatment significantly increased IFN-*γ*+ T cells, while reducing the percentage of CD4+/IL4+ T cells (Figures 3(a) and 3(b)).

Furthermore, DLL treatment increased significantly the percentage of CD8+ T cells in tumor tissues, while having no changes in the percentages of CD4+ T cells and regulatory T cells (Figure 4(a)). The results of immunohistochemistry also confirmed that DLL treatment upregulated the infiltration of CD8+ T cells (Figure 4(b)). As expected, DLL treatment increased the concentration of the IFN-*γ* factor in the tumor tissue (Figure 4(c)). However, DLL treatment did not alter the concentration of IFN-*γ* in the serum (Figure 4(d)). Additionally, DLL treatment significantly upregulated the IFN-*γ* response gene expression, such as Stat1, Irf1, CCL5, CXCL9, and CXCL10 in T cells stored from xenografted tumor tissue (Figure 4(e)). These findings indicate that the antitumor activity of DLL depends on the induction of Th1-type cell-mediated immune responses.

### 3.4. DLL Exerts Antitumor Effects through Mettl3 and Mettl14 and Oxidative Stress

Studies have shown that traditional Chinese medicine exerts antitumor effects through epigenetic effects, and m6A methylation modification plays an important role in cancer immunotherapy, but it was not clear whether DLL-mediated antitumor activity was via m6A methylation modification. We used DLL to treat 3LL cells and detected the expression of key enzymes that regulate m6A methylation modification. DLL significantly inhibited Mettl3 and Mettl14 expression but had no significant effect on the m6A methylase WTAP and the m6A demethylase FTO and ALKBH5 (Figure 5(a)). Western blot results also showed that DLL significantly inhibited the protein levels of m6A methyltransferases Mettl3 and Mettl14 (Figure 5(b)).

RETRACTED

IFN-*γ* can stimulate the production of CCL5, CXCL9, and CXCL10 to enhance antitumor immune response [21]. Our results show that DLL mainly exerted antitumor activity by enhancing the CD8+ T cell recruitment in tumor tissues and the release of IFN-*γ* factors (Figure 4). Stat1, Stat4, Irf1, Irf4, and Irf7 are important transcription factors that regulate the release of cytokines/chemokines. DLL treatment significantly upregulated the levels of Stat1 and Irf1 and the release of cytokines CCL5, CXCL9, and CXCL10 in 3LL cells (Figures 5(a)–5(c)). The balance of oxidation and antioxidation is closely related to the occurrence and development of lung cancer. SOD and GPx are important antioxidative metal enzymes [22, 23]. We tested the level of tumor cell oxidative stress after DLL treatment and found that DLL treatment significantly inhibited the expression of NADPH, SOD1, and GPX and the activity of SOD and GPx, promoted the level of ROS, and reduced the levels of NAD+/NADH and ATP compared with the control (Figures 5(d) and 5(e)).

Given that STAT1 and IRF1 play a key role in IFN-*γ* signal transduction and antitumor effects and DLL administration reduced Mettl3 and Mettl14 expression, while increasing Stat1 and Irf1 expression, we further analyzed whether DLL played a regulatory role on Stat1 and Irf1 through Mettl3 and Mettl14. The results of MeRIP-qPCR demonstrated that DLL intervention dramatically reduced the m6A methylation levels of Stat1 and Irf1 (Figure 5(f)). Ctla4 functioned as a m6A negative control [24].

We also observed that Mettl3 or Mettl14 overexpression significantly attenuated DLL-enhanced Stat1 and Irf1 in 3LL tumor cells (Figures 6(a) and 6(b)), and MeRIP-qPCR results showed that Mettl3 or Mettl14 overexpression significantly enhanced the m6A methylation levels of Stat1 and Irf1 that were reduced by DLL treatment (Figure 6(c)). Mettl3 or Mettl14 overexpression also significantly reduced the concentration of CCL5, CXCL9, and CXCL10 and inhibited ROS accumulation, while increasing SOD concentration in the supernatant of 3LL cell culture (Figures 6(d)–6(f)). These findings suggest that DLL upregulated the expression of Stat1 and Irf1 and enhanced oxidative stress through inhibiting Mettl3 and Mettl14.

RETRACTED

In order to confirm that DLL enhanced T cell activity in tumor-bearing mice through Mettl3 and Mettl14, we purified T cells and cocultured with 3LL cells treated with DLL and/or overexpressed METL3/14 and evaluated T cell proliferation and IFN-*γ* secretion. Compared with the control group, DLL intervention enhanced T cell proliferation, while the overexpression of METL3 and METL14 could significantly reduce the effect of DLL (Figure 6(g)). In addition, DLL treatment significantly upregulated cytokine IFN-*γ* secretion, which was eliminated when METL3/14 was overexpressed (Figure 6(h)). These results indicate that DLL increases the production of cytokines and chemokines through the Mettl3 or Mettl14 pathway.

### 3.5. The Role of DLL Regulating Mettl3, Mettl14, and IFN-*γ* in Tumor Growth Inhibition

IFN-*γ* signaling has a significant impact on the antitumor immune response [25]. We next studied the effect of overexpression of Mettl3 or Mettl14 and anti-IFN-*γ* antibody on the antitumor activity of DLL *in vivo*. The results of in vivo experiments showed that anti-IFN-*γ* antibody administration and overexpression of Mettl3 or Mettl14 enhanced tumor growth, which significantly reversed the antitumor activity of DLL (Figure 7(a)). Further analysis of immune cells in tumor tissues found that overexpression of Mettl3 or Mettl14 and anti-IFN-*γ* antibodies significantly reduced DLL-mediated CD8+ T recruitment (Figures 7(b) and 7(c)) and reduced IFN-*γ* secretion in tumor tissues (Figure 7(d)). In addition, Mettl3 or Mettl14 overexpression significantly inhibited the expression of closely related genes Stat1, Irf1, CCL5, CXCL9, and CXCL10 in the IFN-*γ* pathway (Figures 7(e)–7(i)). Furthermore, Mettl3 or Mettl14 overexpression significantly inhibited the ROS accumulation and increased SOD and GPX levels (Figures 7(j)–7(m)). These results demonstrated that DLL enhanced tumor cell oxidative stress and CD8+ T cell recruitment, ultimately exerting antitumor activity.

## 4. Discussion

Delicaflavone (DLL) is a hydrophobic component extracted from the plant *Selaginella doederleinii* [26]. DLL inhibited lung cancer growth via the endoplasmic reticular stress pathway and Akt/mTOR/p70S6K signaling pathway [6, 20], induced cervical cancer cell apoptosis via the mitochondrial pathway [27], and induced ROS-mediated colorectal cancer cell apoptosis [5]. In this study, we found that DLL inhibited lung cancer growth both *in vitro* and *in vivo*. Furthermore, DLL effectively inhibited tumor growth in immunocompetent mice.

Tumor cell-released immunosuppressive cytokines cause cancer immunotherapy to fail. Some Chinese medicine extracts, such as Trichosanthin, induce immunosuppressive responses [28]. However, no research has been published on the role of DLL in antitumor immunity. We reported for the first time that DLL treatment reduced CD8+ T cell percentage in naive mice. Interestingly, in tumor-bearing mice, we observed that DLL significantly upregulated Th1 cytokine production and enhanced CD8+ T cell infiltration in tumor tissues, thereby enhancing the antitumor immune response.

RETRACTED

Phytochemicals have been demonstrated to have the potential to regulate gene expression by modulating m6A modification. Further mechanism investigation found that DLL significantly inhibited Mettl3 and Mettl14 expression in 3LL cells. Mettl3 or Mettl14 have an oncogene effect on a variety of tumor cells and are closely associated with antitumor immunity [29, 30]. Mettl3 or Mettl14 deficiency inhibited tumor growth in glioblastoma and hepatocellular carcinoma [31–33]. Furthermore, silencing Mettl3 or Mettl14 increased the production of cytokines (such as IFN-*γ* and Cxcl9) and the number of CD8+ T cells in colorectal cancer [19]. In this study, we discovered that Mettl3 or Mettl14 overexpression reversed DLL's antitumor immune activity, as measured by decreased cytokine and chemokine secretion and downregulation of Stat1-Irf1 expression. These findings suggest that DLL activates the antitumor immune system and alters the tumor microenvironment by inhibiting m6A mRNA transferase. As a result, the dynamic imbalance of m6A modification in lung cancer may control immunotherapy response. However, we could not rule out the possibility of writing and erasing specific RNA modifications through enzymatic translocation under various stress conditions.

IFN-*γ* signal activation and IFN-*γ*-Stat1-Irf1 axis are essential to enhance the sensitivity of tumor cells to immunotherapy. Our findings show that anti-IFN-*γ* antibody treatment can eliminate the antitumor activity of DLL. Mechanistically, we revealed that DLL reduced Stat1 and Irf1 m6A modification abundance by inhibiting Mettl3 and Mettl14, thereby upregulating CCL5, CXCL9, and CXCL10 and inducing oxidative stress. Studies have showed that phytochemicals from natural products induce the accumulation of ROS by damaging DNA biomolecules and triggering cell death-related signaling pathways, including m6A modification [34]. m6A alteration is critical in the creation of tumor immune microenvironment variety and complexity in lung cancer [35]. Reactive oxygen species (ROS) can damage lipids, nucleic acids, and proteins, thereby altering their functions. When a balance between the production of ROS and antioxidative defense is disturbed, the state of oxidative stress occurs [36]. ROS might affect the prognosis of cancer patients through immune response and increase the sensitivity of cancer patients to chemotherapy [37]. The traditional Chinese medicine, Jinfukang, induces lung cancer cell apoptosis through the ROS-mediated ATM/ATR-p53 pathway and DNA damage [38]. Arenobufagin caused apoptosis in the non-small-cell lung cancer (NSCLC) cell line A549 by oxidative stress [39]. Our findings suggest that DLL inhibited lung cancer growth by enhancing ROS-mediated cell death.

RETRACTED

CCL5 is a natural adjuvant that can be used to boost antitumor immune responses [40, 41]. This finding explained why the antitumor activity of DLL in nude mice was lower than that in immunocompetent mice. Cxcl9 and Cxcl10 extracellular secretion mediates lymphocyte infiltration into tumors and inhibits tumor growth [42, 43]. The activation of chemokine genes in the tumor environment may result in increased levels of CD8+ T and IFN-*γ* in the tumor. Thus, our research provides solid evidence for the use of DLL as an adjuvant drug for lung cancer immunotherapy.

## 5. Limitations

This study uses a mouse-derived cell line and does not involve the analysis of human samples and cells. There may be differences between mouse-derived cells and human cells. Our follow-up research will continue the investigation. Furthermore, this study did not demonstrate synergy between DLL and existing first-line drugs for lung cancer treatment. If it can be confirmed that DLL can enhance the chemotherapy effect and immunotherapy effect of lung cancer, it will provide a powerful adjuvant drug for lung cancer.

## 6. Conclusion

We found that DLL exerted a tumor suppressor effect by inhibiting m6A transferase and upregulating Stat1 and Irf1 levels to activate antitumor immunity. Our findings provided a potential drug to enhance lung cancer immunotherapy.

## Figures and Tables

**Figure 1:** DLL inhibited 3LL tumor growth both in vitro and in vivo. (a) 3LL tumor cells were treated for 24, 48, and 72 h in a 96-well plate in the presence of different doses of DLL (0, 5, 25, 50, and 100 *μ*g/ml). CCK-8 assay was used to estimate the cell viability. Cell viability was decreased with increased DLL concentration. (b, c) Nude mice (b) and C57BL/6 mice (c) were injected subcutaneously with 5 × 10^4^ 3LL tumor cells per mouse. DLL was injected subcutaneously on day 4 and then once every day for a total of seven injections. Saline was injected subcutaneously as a control. DLL injection significantly inhibited tumor growth in C57BL/6 mice. Data are the mean ± SD from three independent experiments. ^∗∗^*P* < 0.01 and^∗∗∗^*P* < 0.001 by Student's *t*-test, *N* = 6. DLL: delicaflavone.

RETRACTED

**Figure 2:** DLL slightly reduced the percentage of CD8+ T cells and their IFN-*γ* production in naive mice. (a, b) T cells in the LNs (a) and spleen (b) from naive C57BL/6 mice following treatment with DLL or saline were stained with fluorescent antibodies and detected by FACS. DLL treatment reduced the percentage of CD3+/CD8+ T cells and reduced the percentage of CD8+/IFN-*γ*+ cells, while having no effect on the percentage of CD4+/IL4+ T cells and CD4+/IFN-*γ*+ T cells, suggesting that DLL treatment mildly suppressed the initial immune response. Data are the mean ± SD from three independent experiments. ^∗^*P* < 0.05 by Student's *t*-test, *N* = 6. IFN: interferon; LN: lymph node; DLL: delicaflavone.

**Figure 3:** DLL increased the percentage of T cells and the cytokine production in tumor-bearing mice. T cells derived from LNs (a) and spleen (b) of DLL-treated tumor-bearing mice were stained with fluorescent antibodies. Foxp3 and cytokine production of CD4+ and CD8+ T cells were also analyzed by detecting intercellular expression. DLL treatment significantly increased the percentage of CD3+ T cells, CD8+ T cells, and IFN-*γ*+ T cells in the lymph nodes and spleen and decreased the percentage of Treg T cells and CD4+/IL4+ T cells. Data are the mean ± SD from three independent experiments. ^∗^*P* < 0.05 by Student's *t*-test, *N* = 6. LN: lymph node; DLL: delicaflavone.

**Figure 4:** DLL enhances tumor-infiltrating CD8+ T cells and cytokine production. (a) Percentage of tumor-infiltrating T cells and Treg cells was identified by flow cytometry from 3LL tumors as indicated. (b) Representative images of CD8 by IHC staining. Tissue sections from BALB/c mice treated with DLL or saline. Scale bars, 200 *μ*m. DLL treatment significantly increased the percentage of CD8+ T cells in tumor. (c, d) IFN-*γ* production in intratumor (c) and serum (d) from BALB/c mice by ELISA. DLL treatment significantly increased IFN-*γ* in tumor but not in serum. (e) Quantitative RT-PCR was performed to identify transcriptional changes of the IFN-*γ* response gene expression in T cells stored from xenografted tumor tissues. DLL treatment significantly upregulated the levels of Stat1, Irf1, CLL5, CXCL9, and CXCL10 in T cells. Data are the mean ± SD from three independent experiments. ^∗^*P* < 0.05 by Student's *t*-test, *N* = 6. DLL: delicaflavone.

**Figure 5:** DLL reduces Mettl3/Mettl14-mediated m6A modification on Stat1 and Irf1. 3LL cells were treated with DLL or saline. (a) Quantitative RT-PCR was performed to identify mRNA levels of the m6A transferases (left) and the IFN-*γ* response gene expression (right). (b) Western blot analysis of Mettl3, Mettl14, Stat1, and Irf1 in DLL-treated 3LL cells. DLL treatment significantly inhibited Mettl3 and Mettl14 expression, while upregulating Stat1 and Irf1 expression in DLL-treated 3LL cells. (c) CLL5, CXCL9, and CXCL10 production in cell culture supernatant by ELISA. DLL treatment significantly upregulated the levels of CLL5, CXCL9, and CXCL10. (d) Western blot analysis of NADPH, SOD1, and GPX in DLL-treated 3LL cells. DLL treatment significantly inhibited NADPH, SOD1, and GPX expression. (e) The ROS, NAD+/NADH, and ATP levels were measured. DLL treatment significantly promoted the level of ROS and reduced the levels of NAD+/NADH and ATP compared with the control (left). The level of SOD and GPx was measured (right). GAPDH was used as an invariant internal control for calculating protein fold changes. DLL treatment significantly inhibited the activity of SOD and GPx compared with the control. (f) m6A enrichment of Stat1 and Irf1 was examined by m6A RIP-qPCR in control, DLL-treated 3LL cells as indicated. Ctla4 functioned as a m6A negative control. DLL treatment dramatically reduced the m6A methylation on Stat1 and Irf1. Data are the mean ± SD from three independent experiments. ^∗^*P* < 0.05 by Student's *t*-test, *N* = 6. DLL: delicaflavone.

RETRACTED

**Figure 6:** Overexpression of Mettl3 or Mettl14 attenuates DLL-mediated IFN-*γ* response. (a) Mettl3 and Mettl14 expression was upregulated in 3LL cells after infection with Mettl3 or Mettl14 expressing lentivirus. (b) The expression of p-Stat1 (phosphorylated), Stat1, and Irf1 was reduced by infection with Mettl3 or Mettl14 expressing lentivirus in DLL-treated 3LL cells. (c) The m6A modification of Stat1 and Irf1 was upregulated by infection with Mettl3 or Mettl14 expressing lentivirus in DLL-treated 3LL cells evaluated by m6A RIP-qPCR. (d) CLL5, CXCL9, and CXCL10 production in cell culture supernatant was reduced by infection with Mettl3 or Mettl14 expressing lentivirus in DLL-treated 3LL cells evaluated by ELISA. (e) The ROS levels were reduced by infection with Mettl3 or Mettl14 expressing lentivirus in DLL-treated 3LL cells. (f) The level of SOD was increased by infection with Mettl3 or Mettl14 expressing lentivirus in DLL-treated 3LL cells. (g) 3LL cells were cocultured for 4 days with T cells acquired from tumor-bearing mice. The specific proliferation of T cells was measured by BrdU incorporation. The proliferation of T cells was inhibited by Mettl3 or Mettl14 expressing 3LL cells, which was reversed by DLL treatment. (h) The secretion of IFN-*γ* was detected by ELISA in cell culture supernatant that 3LL cells cocultured for 4 days with T cells acquired from tumor-bearing mice. The secretion of IFN-*γ* was reduced by coculturing with Mettl3 or Mettl14 expressing 3LL cells, which was reversed by DLL treatment. Data are the mean ± SD from three independent experiments. ^∗^*P* < 0.05 and^∗∗^*P* < 0.01 by Student's *t*-test, *N* = 6. DLL: delicaflavone.

RETRACTED

**Figure 7:** Overexpression of Mettl3 or Mettl14 attenuates DLL-mediated tumor-infiltrating CD8+ T cells and cytokine production. (a) Mice bearing control and Mettl3 or Mettl14 overexpressed tumors were treated with IFN-*γ* blocking antibody and DLL as indicated. Tumor volume was measured over time points. The inhibitory effects of DLL on tumor growth were reversed by Mettl3 or Mettl14 overexpression or IFN-*γ* blocking antibody treatment. (b) Percentage of tumor-infiltrating T cells and Treg cells were identified by flow cytometry from 3LL tumors as indicated. (c) Representative images of CD8 by IHC staining. Tissue sections from BALB/c mice bearing the indicated treatments. DLL-promoted CD8+ T infiltration was reversed by Mettl3 or Mettl14 overexpression or IFN-*γ* blocking antibody treatment. Scale bars, 200 *μ*m. (d) IFN-*γ* production in intratumor from BALB/c mice by ELISA. DLL-promoted IFN-*γ* secretion was reversed by Mettl3 or Mettl14 overexpression or IFN-*γ* blocking antibody treatment. (e–i) Quantitative RT-PCR was performed to identify transcriptional changes in the IFN-*γ* response gene expression. DLL-enhanced Stat1, Irf1, CLL5, CXCL9, and CXCL10 levels were reversed by Mettl3 or Mettl14 overexpression or IFN-*γ* blocking antibody treatment. (j) The representative images of ROS in tumor. DLL-promoted ROS products were reversed by Mettl3 or Mettl14 overexpression or IFN-*γ* blocking antibody treatment. (k–m) ELISA was performed to measure the concentration of ROS, SOD, and GPX in tumor tissues. DLL-enhanced ROS levels and DLL-reduced SOD and GPX levels were reversed by Mettl3 or Mettl14 overexpression or IFN-*γ* blocking antibody treatment. Data are the mean ± SD from three independent experiments. ^∗^*P* < 0.05 by Student's *t*-test, *N* = 6. DLL: delicaflavone.

## Data Availability

The data that support the findings of this study are available from the corresponding authors upon reasonable request.

## Supplementary Materials

Supplementary Materials Supplementary Table 1: primers used in quantitative polymerase chain reaction.
